The article "Prevalence and Causes of Blindness and Visual Impairment and Their Associated Risk Factors, in Three Tribal Areas of Andhra Pradesh, India" was published in 2014. Journal: PLoS One.

# Prevalence and Causes of Blindness and Visual Impairment and Their Associated Risk Factors, in Three Tribal Areas of Andhra Pradesh, India

**DOI:** 10.1371/journal.pone.0100644

**Published:** 2014-07-09

**Authors:** Nakul Singh, Shiva Shankar Eeda, Bala Krishna Gudapati, Srinivasa Reddy, Pushkar Kanade, Ghanshyam Palamaner Subash Shantha, Padmaja Kumari Rani, Subhabrata Chakrabarti, Rohit C Khanna

**Affiliations:** 1 Biostatistics, Harvard School of Public Health, Boston, Massachusetts, United States of America; 2 Andhra Pradesh Right to Sight Society, Hyderabad, India; 3 School of Optometry and Vision Science, University of New South Wales, Sydney, Australia; 4 Internal Medicine, St. Vincent Charity Medical Center, Cleveland, Ohio, United States of America; 5 Johns Hopkins Bloomberg School of Public Health, Baltimore, Maryland, United States of America; 6 Department of Internal Medicine, Wright Center for Graduate Medical Education, Pennsylvania, United States of America; 7 Brien Holden Eye Research Centre, L.V. Prasad Eye Institute, Banjara Hills, Hyderabad, India; 8 Allen Foster Research Centre for Community Eye Health, GPR International Centre for Advancement of Rural Eye care, L V Prasad Eye Institute, Hyderabad, India; National Eye Institute, United States of America

## Abstract

**Objective:**

To assess the prevalence of blindness and visual impairment (VI), their associated causes and underlying risk factors in three tribal areas of Andhra Pradesh, India and compare this data in conjunction with data from other countries with low and middle income settings.

**Methods:**

Using a validated Rapid Assessment of Avoidable Blindness methodology, a two stage sampling survey was performed in these areas involving probability proportionate to size sampling and compact segment sampling methods. Blindness, VI and severe visual impairment (SVI) were defined as per the WHO guidelines and Indian definitions.

**Results:**

Based on a prior enumeration, 7281 (97.1%) subjects were enrolled (mean age  = 61.0+/−7.9 years). Based on the presenting visual acuity (PVA), the prevalences of VI, SVI and blindness were 16.9% (95% CI: 15.7–18.1), 2.9% (95% CI: 2.5–3.4), and 2.3% (95% CI: 1.9–2.7), respectively. When based on the Pinhole corrected visual acuity (PCVA), the prevalences were lower in VI (6.2%, 95% CI: 5.4–6.9), SVI (1.5%, 95% CI: 1.2–1.9) and blindness (2.1%, 95% CI: 1.7–2.5). Refractive error was the major cause of VI (71.4%), whereas, cataract was the major cause of SVI and blindness (70.3%). Based on the PVA, the odds ratio (OR) of blindness increased in the age groups of 60–69 years (OR = 3.8, 95% CI: 2.8, 5.1), 70–79 years (OR = 10.6, 95% CI: 7.2, 15.5) and 80 years and above (OR = 30.7, 95% CI: 19.2, 49). The ORs were relatively higher in females (OR = 1.3, 95% CI: 1.0, 1.6) and illiterate subjects (OR = 4.3, 95% CI: 2.2, 8.5), but lower in those wearing glasses (OR = 0.2, 95% CI: 0.1, 0.4).

**Conclusions:**

This is perhaps the first study to assess the prevalence of blindness and VI in these tribal regions and the majority of the causes of blindness and SVI were avoidable (88.5%). These findings may be useful for planning eye care services in these underserved regions.

## Introduction

Recent estimates show that there are 324 million people who are either blind or visually impaired in the world and that the burden of blindness and visual impairment (VI) is disproportionately clustered in the developing countries, including India [1]. With 8 million blind people and 62 million VI, India shares almost a quarter of the entire global burden of blindness and VI [1]. Although several prevalence of blindness studies have been reported in Indian populations, [2]–[9] there are limited studies in tribal populations, who are considered the “under-served of the under-served” [10].

India has a large and diverse tribal population, a category formally recognized by the Indian constitution. Tribal communities are characterized by their economic under-development, distinct cultural heritage and geographic isolation [11]. Areas that historically had high tribal populations are formally recognized by the Integrated Tribal Development Agency (ITDA), which aims to develop these tribal areas. ITDA has recently granted funds to implement eye care services in these tribal areas. In order to adequately serve these populations, it was necessary to assess the burden of blindness and VI in these communities, along with their causes.

Earlier we reported the visual outcomes and risk factors for poor outcomes [12]. Herein we report the prevalence of blindness and visual impairment, as well as its causes and their associated risk factors in these three selected tribal areas. Additionally this data was compared with the prevalence and causes of blindness in other countries with low and middle-income settings.

## Methods

The Ethics Committee of the L V Prasad Eye Institute, Hyderabad, India, approved this study and it was conducted in accordance with the tenets of the Declaration of Helsinki.

Prior to undertaking this study, all the procedures were explained in detail to each subject in presence of community heads of the villages. Subsequently, a written consent was obtained from all subjects with minimal level of literacy and thumb impression was obtained from those who did not have a formal education.

There are several areas within Andhra Pradesh (AP) that are formally recognized by the government as tribal areas. Three areas in AP as outlines in our previous study were enumerated [12].

The sampling strategy based on Rapid Assessment of Avoidable Blindness (RAAB) methodology [13] and details of the methodology have been described elsewhere [12]. The definitions of blindness and VI used in the study are both the World Health Organization (WHO) and Indian Ministry of Health (MoH) [14].

The definitions of refractive error, cataract and glaucoma was as defined earlier [12]. Any fundus pathology other than glaucoma was characterized as posterior segment pathology.

Additional information was collected on tribal status and literacy. Illiteracy was defined as self-report of not able to read and write.

Standard training and Inter Observer Variation Test (IOVT) was performed for each of the three teams for measurement of visual acuity (VA), lens examination and causes of blindness and VI to ensure acceptable agreement (Kappa value ≥0.6). IOVT was conducted on 28 subjects by each of the three teams. IOVT for VA testing was conducted on ophthalmic assistants and for clinical findings, on ophthalmologists participating in the survey. IOVT was also done during the course of study for the measurement of VA, lens examination and to study the causes of blindness and VI in 6 preselected clusters (2 in each area). All subjects with PVA <6/18 in either eye, all subjects with previous cataract surgery and 10% of normal subjects were tested by the ophthalmic assistants for VA testing and by ophthalmologist for clinical findings. A total of 114 subjects were tested for IOVT and it showed a kappa value of more than 0.6. Before the start of main study, a pilot study was also done in a rural area and a total of 51 persons were examined.

All subjects aged ≥50 years in the population in the research area, residing in the village for the last 6 months and willing to give informed consent were selected for the study. All protocols followed the standard RAAB manual [13].

STATA version 11 was used to analyze the data [15]. The prevalence of blindness, SVI and VI by presenting and pinhole-corrected visual acuity were calculated. Risk factors for VI and <6/60 (blindness using the Indian definition) were assessed using univariable and multivariable logistic regression. Multi-collinearity between variables was assessed looking at the variance inflation factor and calibration of the models were assessed by the Hosmer-Lemeshow test for goodness of fit [16].

## Results

Overall 7281/7500 (97.1%) individuals were examined. Among the remaining, 154 (2.1%) were not available, 49 (0.7%) refused and 16 (0.2%) were unable to communicate. There was no significant difference in mean ages (p = 0.46) and gender (p = 0.3) between participants and non-participants (Table 1).

**Table 1:** Baseline characteristics of participants and non-participants.

Subjects	Total	Participants	Non-participants
	N (%)	N (%)	N (%)
**Age group**			
50–59	3296 (44.0)	3216 (44.2)	80 (36.5)
60–69	2877 (38.4)	2770 (38)	107 (48.9)
70–79	1082 (14.4)	1058 (14.5)	24 (11.0)
> = 80	245 (3.3)	237 (3.3)	8 (3.7)
**Mean age (SD)**	61.0 (7.9)	61.0 (7.9)	61.4 (7.2)
**Gender**			
Male	3324 (44.3)	3219 (44.2)	105 (48.0)
Female	4176 (55.7)	4062 (55.8)	114 (52.1)
Literacy			
Literate	873 (11.6)	866 (11.9)	7(3.20)
Illiterate	6627 (88.4)	6415 (88.1)	212 (96.8)
**Tribal versus non-tribal**			
Non Tribal	4547 (60.6)	4429 (60.8)	118 (53.9)
Tribal	2953 (39.4)	2852 (39.2)	101(46.1)

SD: Standard Deviation.

Based on PVA, the prevalence of VI was 16.9% (95% CI: 15.7–18.1), SVI was 2.9% (95% CI: 2.5–3.4), and blindness was 2.3% (95% CI: 1.9–2.7). The prevalence of blindness as per the Indian definition was 5.2 (95% CI: 4.6–5.9). Based on PCVA, the prevalence of VI was 6.2% (95% CI: 5.4–6.9), SVI was 1.5% (95% CI: 1.2–1.9), and blindness was 2.1% (95% CI: 1.7–2.5). The prevalence of blindness as per the Indian definition was 3.6 (95% CI: 3.1–4.2) (Table 2)

**Table 2:** Prevalence of Blindness, SVI and VI based on presenting and Pinhole-corrected visual acuity.

Presenting visual acuity							
Total		VI (<6/18–6/60)		SVI (<6/60–3/60)		Blindness (<3/60)	
	N	N	% (95% CI)	N	% (95% CI)	N	% (95% CI)
**Male**	3219	579	18.0(16.5–19.5)	94	2.9 (2.3–3.5)	54	1.7 (1.2–2.2)
**Female**	4062	649	16.0(14.5–17.5)	119	2.9 (2.3–3.5)	114	2.8 (2.3–3.3)
**Total**	7281	1228	16.9(15.7–18.1)	213	2.9 (2.5–3.4)	168	2.3(1.9–2.7)

Pinhole corrected visual acuity (pin-hole)							
Total		VI (<6/18–6/60)		SVI (<6/60–3/60)		Blindness (<3/60)	
	N	N	% (95% CI)	N	% (95% CI)	N	% (95% CI)
**Male**	3219	218	6.8(5.7–7.9)	47	1.5 (1.0–1.9)	49	1.5(1.0–2.0)
**Female**	4062	230	5.7(4.8–6.5)	65	1.6 (1.1–2.1)	104	2.6 (2.1–3.0)
**Total**	7281	448	6.2(5.4–6.9)	112	1.5 (1.2–1.9)	153	2.1 (1.7–2.5)

VI: Visual Impairment; SVI: Severe Visual Impairment; CI: Confidence Interval.

Based on PVA and PCVA, the odds of VI and blindness (Indian definition) increased with age and illiteracy. Additionally, the odds of blindness were significantly higher in female subjects. Based on PVA, odds of VI and blindness were lower in those wearing glasses, and Area 3 had lower odds of VI (Tables 3 and 4).

**Table 3:** Presenting Visual Acuity: Risk factors for VI, SVI and blindness.

	VI	Blindness+ SVI
	Multivariate OR (95% CI)	Multivariate OR (95% CI)
**Age group**		
50–59	Ref	Ref
60–69	**2.84(2.4,3.35)**	**3.77(2.77,5.13)**
70–79	**4.80(3.94,5.84)**	**10.56(7.22,15.45)**
80+	**7.27(5.14,10.3)**	**30.72(19.24,49.04)**
**Gender**		
Male	Ref	Ref
Female	0.93(0.81,1.07)	1.28(1.01,1.61)
Literacy		
**Literate**	Ref	Ref
Illiterate	1.71(1.29,2.27)	4.34(2.23,8.45)
**Tribal status**		
Non–tribal	Ref	Ref
Tribal	1.00(0.82,1.22)	1.16(0.86,1.56)
**Area**		
1	Ref	Ref
2	0.84(0.68,1.05)	0.72(0.5,1.03)
3	**0.74(0.58,0.95)**	0.97(0.7,1.35)
**Use of glasses**		
No	Ref	Ref
Yes	**0.71(0.56,0.91)**	**0.21(0.12,0.38)**
**Goodness of fit ‘p’ value**	0.302	0. 6597

VI: Visual Impairment; SVI: Severe Visual Impairment; CI: Confidence Interval; Ref: Reference group; OR: Odds Ratio.

**Table 4:** Pinhole Corrected Visual Acuity: Risk factors for VI, SVI and Blindness.

	VI	Blindness+ SVI
	Multivariate OR (95% CI)	Multivariate OR (95% CI)
**Age group**		
50–59	Ref	Ref
60–69	**3.35(2.5,4.48)**	**3.18(2.14,4.72)**
70–79	**6.53(4.72,9.05)**	**9.34(5.92,14.72)**
80+	**10.21(6.64,15.72)**	**22.89(13.35,39.25)**
**Gender**		
Male	Ref	Ref
Female	0.88(0.71,1.09)	1.45(1.11,1.88)
**Literacy**		
Literate	Ref	Ref
Illiterate	**2.18(1.46,3.25)**	**4.31(1.84,10.09)**
**Tribal status**		
Non-tribal	Ref	Ref
Tribal	1.08(0.8,1.45)	1.37(0.97,1.92)
**Area**	0.0063	0.2471
1	Ref	Ref
2	0.71(0.5,1.01)	0.75(0.50,1.13)
3	1.31(0.95,1.79)	1.05(0.73,1.53)
**Goodness of fit ‘p’ value**	.1602	.7054

VI: Visual Impairment; SVI: Severe Visual Impairment; CI: Confidence Interval; Ref: Reference group; OR: Odds Ratio.

Refractive error (including uncorrected aphakia) was the major cause of VI (71.4%) and cataract was major cause of SVI and blindness (70.3%). Together, posterior segment disorders (including glaucoma) caused 4.2% of VI and 11.6% SVI and blindness. (Table 5)

**Table 5:** Causes of VI, SVI and blindness.

Cause	VI N (%)	SVI +Blindness N (%)
**Refractive Error**	869 (70.8)	36 (9.5)
**Cataract untreated**	287 (23.4)	268 (70.3)
**Aphakia uncorrected**	7 (0.6)	10 (2.6)
**Surgical Complication(s)**	11 (0.9)	4 (1.1)
**Phthisis**	0 (0.0)	4 (1.1)
**Corneal scar**	2 (0.2)	15 (3.9)
**Glaucoma**	8 (0.7)	8 (2.1)
**Other posterior segment diseases**	44 (3.5)	36 (9.5)
**Total**	1228	381

VI: Visual Impairment; SVI: Severe Visual Impairment.

There was no significant difference in the use of glasses between males and females (p = 0.273). However, use of glasses was significantly less likely in tribal subjects than non-tribal subjects (p<0.001), illiterate than literate subjects (p<0.001) and subjects residing in areas 2 and 3 to those residing in Area 1 (p<0.001).

## Discussion

This study was designed specifically to report the prevalence of blindness and VI in tribal areas in the state of AP and the observed prevalence compares favorably to other populations in India and in neighboring countries found in the last decade. Using the same definition, the observed prevalence of blindness in this study is similar to the other studies in India [2], [4], [9] and neighbouring countries like Nepal [17], [18], Bangladesh [19] and Pakistan [20]. (Table 6) However, the prevalence is much lower than many other studies reported in India [3], [6]–[8] and countries like Nepal [21] and Myanmar [22]. The observed prevalence is also lower than the two reported studies from tribal areas of India [10] and Pakistan [23] and was higher that some other studies from Nepal [24], Pakistan [25] and China [26] (Table 6). The potential causes for these observed differences are many; they may reflect regional differences in terms of availability of services, time periods when the studies were conducted, age groups included in the population, cultural beliefs for health-promoting behaviors, or, most simply, sampling variation in these studies. For instance, the national prevalence was a pooled prevalence from 16 districts of 15 states and the prevalence of individual districts was not reported [8]. This might obscure the variability within the regions. Similarly, the study in Bharatpur, Rajasthan was conducted a decade earlier than this study, and the differences in prevalence might be a reflection of the changing trends of blindness over time [6]. Additionally, we observed that the prevalence of presenting VI was 16.9% (95% CI: 15.7–18.1), which was comparable to tribal region of Maharashtra [10], the Lumbini zone and Chetwan district of Nepal [18], and the national survey [8]. When compared to other studies done in India and elsewhere, the prevalences were highly variable [2]–[4], [6], [7], [9], [17], [19], [21], [24]–[26] (Table 6), which could be due to the same reasons mentioned above.

**Table 6:** Prevalence of blindness, SVI and VI in different studies in India and neighboring countries.

Country (Year of survey)	Region	Age group	Number examined (%)	Blindness (95% CI)	SVI (95% CI)	VI (95% CI)
**India (1998) ** [6]	Rajasthan (Bharatpur)	> = 50	4284 (90.6)	8.9 (7.2–10.5)	3.1 (2.3–3.8)	24.3 (23.0–25.6)**
**India (1999) ** [9]	Rural South India (Sivaganga)	> = 50	4642 (91.4)	4.0 (3.5–4.5)	2.0 (1.4–2.7)	28.5 (27.2–29.8)**
**India (2007) ** [8]	National (16 districts of 15 states)	> = 50	40447 (94.7)	3.6 (3.3–3.9)	4.4 (4.1–4.8)	16.8 (16.0–17.5)
**India (2007) ** [7]	Gujarat	> = 50	4738 (91.9)	4.3 (3.5–5.1)	2.6 (1.8–3.4)	29.3 (27.5–31.2)
**India (2011) ** [2]	Karnataka (Kolar)	> = 50	2907 (95.3)	3.9 (2.74–5.1)	3.5 (2.49–4.46)	10.4 (8.77–12.08)
**India (2009) ** [10]	Maharashtra (Nandurbar)	> = 50	2004 (87.2)	1.87 (1.32–2.42)	6.72 (5.7–7.74)	19 (17.4–20.6)
**India (2010) ** [4]	Prakasam Weavers South	> = 40	2848 (94)	2.9 (2.3–3.5).	NA	9.4 (8.3–10.5)
**Nepal (2002) ** [24]	Gandaki Zone	> = 45	5002 (85.3)	1.4 (1.1–1.8) **	1.2 (0.9–1.5)**	8.9 (8.1–9.7)**
**Nepal (2006) ** [18]	Lumbini Zone & Chitwan District	> = 50	5138 (87)	2.3 (1.7–2.8)	2.3 (1.5–3.2)	16 (15.0–17.0) **
**Nepal (2006) ** [21]	Rautahat District	> = 50	4717 (85.3)	6.9 (5.5–8.3)	10.5 (9.3–11.8)	25.6 (24.4–26.9) **
**Nepal** * [17]	Karnali Zone	> = 50	1174 (97.8)	3.4 (2.4–4.4)	2.1 (1.4–3.1) **	9.7 (8.1–11.5) **
**Bangladesh (2005) ** [19]	Satkhira District	> = 50	4868 (91.9)	2.9(2.4–3.5)	1.6(1.2–2.0)	8.4(7.5–9.3)
**Pakistan** * [23]	Tribal Area (Orakazi Agency)	> = 50	1549 (96.8)	5.9 (4.7–7.0)	NA	NA
**China (2006) ** [27]	Kunming	> = 50	2588 (93.8)	2.7 (2.1–3.4) **	3 (2.2–3.8)	9.1 (7.5–10.7);
**China (2006) ** [26]	Rural (9 Provinces)	> = 50	45747 (90.8)	2.29 (2.08–2.50)	1.36 (1.17–1.56)	9.39 (8.99–9.80)
**Myanmar (2005) ** [22]	Meiktila (Rural Myanmar)	> = 40	2076 (83.6)	8.1(6.5–9.9)	NA	32.9 (27.7–38.1)

*: Year of study not available; CI: Confidence Interval;

**: Confidence Interval calculated using binomial proportions; SVI: Severe Visual Impairment; VI: Visual Impairment; NA: Data not available.

Both univariable and multivariable analysis indicated older age to be a major risk factor for VI and blindness in PVA and PCVA. This is consistent to findings observed in other studies from India and adjoining developing nations [4], [6]–[10], [17], [18], [21], [22], [24], [26], [27] (Table 7). Additionally, females were more likely to be blind by PVA (OR 1.28, 95% CI: 1.01–1.61) and PCVA (OR 1.45, 95% CI: 1.11–1.88). These findings are however are partially consistent with some studies [4], [6], [8], [17], [21], [26], but not in others [7], [9], [10], [24] (Table 7). While this disparity may be grossly attributed to different social experiences and/or different barriers to accessing eye care services, further studies are needed to understand the underlying causes.

**Table 7:** The risk factors for Blindness and VI based on presenting visual acuity across different studies in India and neighbouring countries.

Country (Year)	Region	Age group	OR (95% CI)	OR (95% CI)	OR (95% CI)	OR (95% CI)
			Age	Female gender	Illiteracy	Rural location
**India (2001) ** [6]	Rajasthan (Bharatpur)	50–59	Ref	1.6 (1.3–2)	2.8 (2.0–3.7)	1.7 (1.0–2.8)
		60–69	3.8 (2.8–5.1)			
		> = 70	12.8 (9.6–17.1)			
**India (2002) ** [9]	Rural South India (Sivaganga)	50–59	Ref	1.1(0.8–1.4)	2.6(1.7–4.0)	1.0 (0.6–1.7)
		60–69	2.6(1.9–3.6)			
		> = 70	5.6(4.0–8.0)			
**India (2008) ** [8]	National (16 districts of 15 states)	50–54	Ref	1.56 (1.45–1.72)	NA	1.2 (1.1–1.33)
		55–59	1.91 (1.54–2.38)			
		60–64	3.65 (2.99–4.45)			
		65–69	4.92 (4.03–6.01)			
		> = 70	7.42 (6.07–9.06)			
**India (2010) ** [7]	Gujarat	50–59	Ref	0.92(0.68–1.23)∧	0.22(0.16–0.31)*	0.7 (0.41–1.2)$
		60–69	2.7(2–3.6)			
		> = 70	5.9(4.2–8.3)			
India (2012) [10]	Maharashtra (Nandurbar)	NA	+	1.5(.75–3.75)	NA	NA
**India (2013) ** [4]	Prakasam Weavers South	40–49	Ref	1.3(1.0–1.7)	1.7 (1.3–2.2)*	NA
		50–59	3.5 (2.5–5.2)			
		60–69	8.7(5.9–12.7)			
		> = 70	22.4(15.0–33.5)			
**Nepal (2006) ** [24]	Gandaki Zone	45–49	Ref	1.1 (0.8–1.7)	3.5(1.7–7.1)	NA
		50–60	1.7(0.6–4.9)			
		61–70	4.7(1.8–12.4)			
		>70	24.0(9.5–60.3)			
**Nepal (2009) ** [18]	Lumbini Zone & Chitwan District	50–59	Ref	NA	2.9(1.6–5.1)	NA
		60–69	3.2(2.2–4.6)			
		> = 70	6.1(4.1–9.1)			
**Nepal (2010) ** [21]	Rautahat District	50–59	Ref	1.4(1.1–1.7)	2.0(1.5–2.8)	NA
		60–69	2.7(2.3–3.1)			
		> = 70	6.6 (5.4–8.0)			
**Nepal (2012) ** [17]	Karnali Zone		+	++	NA	NA
**China (2008) ** [27]	Kunming		+	NA	NA	2.9 (1.5–5.3)
**China (2010) ** [26]	Rural (9 Provinces)	50–59	Ref	1.50 (1.31–1.72)	#0.78 (0.62–0.98)*	NA
		60–69	2.61(2.03–3.35)		&0.6(0.43–0.86)*	
		70–79	8.96(6.95–11.6)			
		> = 80	29.4(22.2–39.0)			
**Myanmar (2007) ** [22]	Meiktila (Rural Myanmar)	40–49	Ref			
		50–59	2.8(1.3–5.2)	1.3 (0.8–1.8)	1.4 (1.0–2.0)	NA
		60–69	6.5(3.4–12.3)			
		> = 70	11.9(6.3–22.5)			

OR: Odds Ratio; Ref: Reference Group; CI: Confidence Interval;

∧: Reference group: Female;

*Reference group: Illiterate;

$ : Reference group: Rural location;

# : Primary education;

& : Secondary education;

+: Higher with increasing age (Odds ratio and 95% CI not available);

++: Higher in females (Odds ratio and 95% CI not available).

Illiteracy was a significant risk factor for blindness and VI, based in PVA and PCVA. This seemed to be a general phenomemenon as observed in other studies [4], [6], [7], [9], [18], [21], [22], [24], [26] (Table 7). Furthermore, we also observed that illiterate subjects were less likely to use glasses that is indicative of a major barrier to accessing eye care services. Whether this is due to poverty or lack of knowledge needs further exploration. It may be recommended that community programs should include illiteracy as a major consideration when planning for outreach activities.

Based on the PVA, the odds of VI was lower in Area 3 in a multivariable analysis. According to local sources, non-tribal subjects migrate to tribal areas to enjoy government-mandated benefits, and they preferentially inhabit areas with burgeoning local economies. Each area varied significantly with respect to the fraction of tribal population and literacy rates within it (p value <0.001) and subjects in Area 3 had significantly higher literacy rates and a lower tribal population compared to other two areas (data not shown). Altogether, these findings indicate that Area 3 has possibly developed the most of the three areas, resulting in better quality of available and accessible services as compared to the other areas. Similarly, those wearing glasses were also at lower risk of blindness and VI based on PVA.

Interestingly, the ‘tribal’ status was not a risk factor for either VI or blindness by any definition indicating that these populations did not face any specific health disparity compared to the ‘non-tribes’. The poor eye health appeared to be characteristic of the areas sampled and not restricted to any specific group of people (i.e. tribal or non tribal). Our findings could be further explained by the fact that both the tribal people and non-tribal people intermix in their daily life and hence, differences in lifestyle or behaviors that leading to a health disparity was unlikely.

While there has been substantial achievements in combating cataract and refractive error-related blindness due to planned eye care services, they still continue to be a major cause of blindness and VI in India and other developing countries (Table 8). The most sobering finding of this study, however, was that 82.4% of the presenting cases of blindness were treatable (untreated cataract, uncorrected aphakia, refractive error) and 6.1% preventable (corneal scars, surgical complications and phthisis). Moreover, we found that 11.6% of blindness was caused by posterior segment disorders (including glaucoma). This is consistent with some of the recent studies from India that exhibited an increase in the prevalence of posterior segment disorders [2], [7]. This fraction is fairly substantial, and it highlights the importance of a dilated fundus examination to assess the cause of blindness in populations.

**Table 8:** Causes of blindness, SVI and VI in different studies in India and neighbouring countries.

Country (Year)	Region	Causes of blindness (%)	Causes of SVI (%)	Causes of VI (%)
India (2001) [6]	Rajasthan (Bharatpur)	Cataract (67.5) and uncorrected aphakia including RE (18.4) in at least one eye	NA	NA
India (2002) [9]	Rural South India (Sivaganga)	Cataract (69.4), RE including uncorrected aphakia (35.6) in one or both eyes*	-	NA
India (2008) [8]	National (16 districts of 15 states)	Cataract (77.5)*	-	Cataract (58.1), RE (32.9)
India (2010) [7]	Gujarat	Cataract (82.6), posterior segment disease (8.9)*	-	Cataract (50.3), RE (35.4)
India (2012) [2]	Karnataka (Kolar)	Cataract (74.6), posterior segment (8.8)	Cataract (73.3), RE (11)	RE (56.1), cataract (35.3)
India (2012) [10]	Maharashtra (Nandurbar)	Cataract (76)	NA	NA
India (2013) [4]	Prakasam Weavers South	Cataract (62.6), RE (20.6)	NA	RE (73.2), cataract (18.6)
Nepal (2006) [24]	Gandaki Zone	Cataract (64.5), RE (13.2)	NA	NA
Nepal (2009) [18]	Lumbini Zone and the Chitwan District	Cataract (48.1); RE (31.4), retinal disorder (4), corneal opacity (3.8)	NA	NA
Nepal (2010) [21]	Rautahat District	Cataract (85.9), RE (7.3)	NA	NA
Nepal (2012) [17]	Karnali Zone	Cataract (67.5)	Cataract (96)	RE (36.8), cataract (58.8)
Bangladesh (2006) [19]	Satkhira District	Cataract (79.0), posterior segment (13.3)	Cataract (78.2), posterior segment (15.4)	RE (52.9), cataract (41.9)
Pakistan (2006) [23]	Tribal Area (Orakazi Agency)	Cataract (82.4)	NA	RE (83.3)
China (2008) [27]	Kunming	Cataract (63.2), trachomatous scar (14.7), glaucoma (7.4)	Cataract (71.4); other posterior segment (7.8)	Cataract (51.7), RE (36)
Myanmar (2007) [22]	Meiktila (Rural Myanmar)	Cataract (53.0) angle closure glaucoma (9.6)	NA	NA

*: For both Blindness and Severe Visual Impairment; RE: Refractive error; SVI: Severe Visual Impairment; VI: Visual Impairment; NA: Data not available.

The major strengths of this study pertains to the fact that it adhered to the RAAB methodology, and had a very high response rate (97.1%). One of the methodological weaknesses of the study was that VI / blindness was determined based on visual acuity and visual fields defects were not included. This may potentially underestimate the prevalence of VI / blindness. Similarly, the prevalence and causes of blindness and VI in those below 50 years could not be estimated. Also, as age and gender were not adjusted for prevalence estimates, it is possible that there could be demographic differences from other studies. As the RAAB methodology assigns primary cause of vision loss to the disorder that can be most easily treated, this study is likely to underestimate the presence of co-morbid causes of vision loss. Additionally, subjects who were illiterate participated in the study at lower rates than literate subjects, suggesting that our estimate of prevalence of blindness is an underestimate. This bias is mitigated by the fact that the study had a very high response rate (97.1%), which is a major strength of this study.

Nevertheless, this study provides an overview for understanding the burden and distribution of blindness and VI and their associated risk factors in these underserved areas. Further research should be aimed at analyzing the issues underlying patients' attitudes, availability, accessibility and affordability of services that affect blindness and VI in these communities.
